The article "Nogo-C Inhibits Peripheral Nerve Regeneration by Regulating Schwann Cell Apoptosis and Dedifferentiation" was retracted in 2025. Reason: concerns about the images.

# Nogo-C Inhibits Peripheral Nerve Regeneration by Regulating Schwann Cell Apoptosis and Dedifferentiation

**DOI:** 10.3389/fnins.2020.616258

**Published:** 2021-01-21

**Authors:** Bo Jia, Wei Huang, Yu Wang, Peng Zhang, Zhiwei Wang, Ming Zheng, Tianbing Wang

**Affiliations:** ^1^Trauma Medicine Center, Peking University People’s Hospital, Beijing, China; ^2^Key Laboratory of Trauma and Neural Regeneration (Peking University), Beijing, China; ^3^National Center for Trauma Medicine of China, Beijing, China; ^4^Department of Physiology and Pathophysiology, Health Science Center, Peking University, Beijing, China

**Keywords:** Nogo-C, Schwann cells, apoptosis, dedifferentiation, peripheral nerve regeneration

## Abstract

While Nogo protein demonstrably inhibits nerve regeneration in the central nervous system (CNS), its effect on Schwann cells in peripheral nerve repair and regeneration following sciatic nerve injury remains unknown. In this research, We assessed the post-injury expression of Nogo-C in an experimental mouse model of sciatic nerve-crush injury. Nogo-C knockout (Nogo-C^–/–^) mouse was generated to observe the effect of Nogo-C on sciatic nerve regeneration, Schwann cell apoptosis, and myelin disintegration after nerve injury, and the effects of Nogo-C on apoptosis and dedifferentiation of Schwann cells were observed *in vitro*. We found that the expression of Nogo-C protein at the distal end of the injured sciatic nerve increased in wild type (WT) mice. Compared with the injured WT mice, the proportion of neuronal apoptosis was significantly diminished and the myelin clearance rate was significantly elevated in injured Nogo-C^–/–^ mice; the number of nerve fibers regenerated and the degree of myelination were significantly elevated in Nogo-C^–/–^ mice on Day 14 after injury. In addition, the recovery of motor function was significantly accelerated in the injured Nogo-C^–/–^ mice. The overexpression of Nogo-C in primary Schwann cells using adenovirus-mediated gene transfer promoted Schwann cells apoptosis. Nogo-C significantly reduced the ratio of c-Jun/krox-20 expression, indicating its inhibition of Schwann cell dedifferentiation. Above all, we hold the view that the expression of Nogo-C increases following peripheral nerve injury to promote Schwann cell apoptosis and inhibit Schwann cell dedifferentiation, thereby inhibiting peripheral nerve regeneration.

## Background

Peripheral nerve injury is a common type of trauma, leading to limb paralysis and limited activity, which may impose a heavy social and economic burden on patients (Abrams and Widenfalk, 2005; Hoke, 2006; Navarro et al., 2007). How to improve the repair of peripheral nerve injury is the focus of clinical and basic research.

Schwann cells play a central role (Huang et al., 2016) in nerve regeneration; they undergo cell reprogramming during Wallerian degeneration (Armstrong et al., 2007; Campana, 2007; Webber and Zochodne, 2010; Allodi et al., 2012) and transform from mature and differentiated myelinating Schwann cells into repairing Schwann cells (Arthur-Farraj et al., 2012, 2017; Jessen and Arthur-Farraj, 2019). In this process, Schwann cells reverse their myelin differentiation. Their characterizing molecules before myelin formation, including L1, NCAM, p75NTR, and glial fibrillary acidic protein (GFAP) and many others, are upregulated. While a large number of genes related to myelination are downregulated, including P0, myelin basic protein (MBP), and membrane associated proteins such as myelin associated glycoprotein (MAG) and periaxin. This type of Schwann cell plays an important role in promoting axonal regeneration. They release cytokines to recruit macrophages and activate the intrinsic demyelination process (which is believed to be the leading cause of demyelination 5–7 days after the injury) (Hirata and Kawabuchi, 2002; Rotshenker, 2011; Vidal et al., 2013). In the first phase of myelin clearance, the Schwann cells break down 40–50% of the myelin during the first 5–7 days after injury. Recently demonstrated that Schwann cells use autophagy to degrade myelin after nerve transection. Subsequently, macrophages that invade injured nerves play the major role in myelin breakdown by phagocytosis in conjunction with antibodies and complement (Gomez-Sanchez et al., 2015; Brosius Lutz et al., 2017). Therefore, Schwann cells with phenotypic transition after nerve injury are involved in the repair of injured nerves via various pathways.

Furthermore, axonal transection leads to neuregulin loss, which is associated with massive Schwann cell apoptosis, and the up-regulation of the apoptosis-inhibiting gene, bcl-2, in Schwann cells reduces apoptosis of Schwann cells after trophic factor withdrawal (Grinspan et al., 1996; Trachtenberg and Thompson, 1996).

Schwann cells participate in peripheral nerve injury repair through cellular dedifferentiation and apoptosis. Therefore, it is important to explore the molecular mechanisms regulating Schwann cell dedifferentiation and apoptosis after nerve injury to provide an in-depth understanding of peripheral nerve repair mechanisms to reveal possible intervention targets.

Nogo is a major inhibitor of CNS axonal regeneration. The Nogo gene family consists of three members, Nogo-A, Nogo-B, and Nogo-C. Nogo-A is located in the CNS and strongly inhibits axonal regeneration (Brosamle et al., 2000; Petrinovic et al., 2010). Nogo-B, a spliced variant of Nogo-A, is widely expressed in all body tissues. Nogo-B is highly expressed in Schwann cells in the local lesions after peripheral nerve injury, mediating Schwann cell apoptosis after peripheral nerve injury, and is regulated by through caspase7 (Schweigreiter et al., 2007). Nogo-C, with a unique sequence at the N-terminus, is distributed in all tissues. Nogo-C promotes liver cancer cell apoptosis and plays an important role in cardiomyocyte apoptosis and fibrosis after myocardial infarction. Elevated expression of Nogo-C and its inhibitory effect on axonal regeneration have been observed in the peripheral nervous system, although the mechanism remains unclear. Using a mouse model, we aimed to understand the role of Nogo-C in regeneration after neuronal injury.

In this study, we aim to reveal the novel mechanism of peripheral nerve injury repair by studying the influence of Nogo-C on peripheral nerve injury, providing a potential new target for quick repair of injured peripheral nerves in clinical practice.

## Materials and Methods

### Ethics Statement

This study was conducted in accordance with the guidelines for the care and use of laboratory animals of the Chinese Association of Laboratory Animal Sciences (ethical approval number 2017PHC065). All animal handling procedures were approved by the Animal Protection Committee of Peking University Health Science Center and every effort was made to minimize the suffering of animals.

### Generation of Nogo-C Knockout Mouse

Nogo-C knockout mice (Nogo-C^–/–^) were generated by TALEN technique with C57BL/6 background. Just as reported (Weng et al., 2018), eight base pairs of exon 1c, the specific exon for Nogo-C, were chopped to induce a frame-shift mutation, resulting in a truncated protein, which may be subject to non-sense mediated decay.

### Mouse Model

Nogo-C knockout mice (Nogo-C^–/–^) were constructed using C57BL/6 mice using the TALEN technique. A mouse sciatic nerve crush injury experimental model was established using 8–12 weeks old male WT C57BL/6 and Nogo-C^–/–^ mice. Mice were anesthetized by intraperitoneal (i.p.) injection of sodium pentobarbital (60 mg/kg). For the experimental (right) side, an oblique incision of about 0.8 cm was made on the hip and the sciatic nerve was exposed and wrapped with a glove as a protection strip at the lower edge of the piriformis, then clamped with a pair of vessel forceps for 30 s before releasing. For the control (left) side, only the sciatic nerve was exposed. All incisions were rinsed and sutured. Postoperative ceftriaxone sodium (0.2 ml intramuscular injection in the gluteus maximus) was given for antibiotic treatment and tramadol (10–30 mg/kg, i.p., q8–12 h for three consecutive days) for analgesia.

### Walking Trajectory Analysis

Pre- and post-operative footprint analysis was performed for all mice according to methods previously reported (Buttner et al., 2018), and SFI was calculated. Briefly, the SFI of both the injured side (E) and the uninjured side (N) of the paw was calculated using measures of print length (PL) mediary toe-spread (IT) and inter-toe-spread (TS), based on the formula:

SFI=-38.3[(EPL-NPL)/NPL]+109.5[(ETS-NTS)/NTS]+13.3[(EIT-NIT)/NIT]-8.8

### Semi-Thin Section

The distal sciatic nerve was removed and placed in 2.5% glutaraldehyde for 4°C overnight. Before slicing, the nerve was placed in 1% osmium tetroxide and fixed for 2 h, then dehydrated with alcohol and embedded in Epon. The 0.5 μm semi-thin section 3–5 mm distal to the lesion was examined by a light microscope equipped with a digital camera.

### Transmission Electron Microscopy (TEM)

The nerve tissue was fixed with 2% glutaraldehyde in sodium dimethylarsenate buffer (0.1 M, pH 7.2) overnight at 4°C and then fixed with 1% osmium tetroxide solution for 1 h. Digital images were acquired with a JEM-1230 high contrast TEM and soft scan imaging system (JEOL, Tokyo, Japan).

### Culture of Schwann Cells

Sciatic nerves were removed from Sprague-Dawley rats 1–2 days after birth and washed in HBSS solution, as previously reported (Tao, 2013; Monje, 2018) (Gibco; Thermo Fisher Scientific, Waltham, MA, United States). These nerves were digested with 0.2% type I collagenase (Gibco) for 30 min at 37°C, followed by 0.25% trypsin (Gibco) for 10 min, and aspirated with 18 G and 21 G needles. The supernatant was collected and centrifuged. Cells were seeded in a Poly-D-Lysine (Gibco)-pretreated culture dish and cultured for 24 h. The medium was replaced with fresh medium containing 10 μM Ara-C (Sigma, St. Louis, MO, United States) and cultured for 3 days to suppress the growth of fibroblasts. Replace the medium containing Ara-C with basic medium and culture 3 more days. Remove fibroblasts using anti-Thy1.1 antibody and rabbit complement (Merck Millipore, Darmstadt, Germany). The medium was replaced with complete medium supplemented with 2 μM forskolin (Sigma) and 10 ng/ml EGF-D (R&D Systems, Minneapolis, MN, United States).

### Construction of Plasmids and Adenovirus

Adenovirus was constructed, as described previously (Jia et al., 2016). Briefly, the amplified product of Nogo-C was inserted into pENTR/TEV/D-TOPO vector (Invitrogen), and constructed product was recombined with pAd/CMV/V5-DEST vector (Invitrogen). Adenovirus was produced with Adenoviral Expression System (Invitrogen) and purified using Vivapure Adeno-PACK Kit (Sartorius, Göttingen, Germany).

### Western Blot

Total protein was extracted from Schwann cells or mouse sciatic nerve with RIPA lysis buffer (Thermo Fisher Scientific) containing protease inhibitor cocktail (Sigma). Total protein concentration was measured using the BCA assay (Pierce, Rockford, IL, United States). Total protein was separated by SDS-PAGE and transferred to a PVDF membrane (Merck Millipore). The membrane was incubated with anti-Nogo-C (Abmart, Shanghai, China), β-actin, Krox-20 (Abcam, MA), and c-Jun, GFAP bcl2 or BAX (CST, United States) primary antibodies. Next, goat anti-rabbit IgG, goat anti-mouse IgG (Biodragon, Beijing, China), or mouse anti-rabbit IgG LCS (Abbkine, Wuhan, China) secondary antibodies were incubated. Immunoblotting was assessed using the Chemi Doc XRS + imaging system (Bio-Rad, Redmond WA, United States).

### RT-PCR

Total RNA was extracted from the sciatic nerve using Trizol (Invitrogen) reagent, according to manufacturer’s instructions. RNA samples were reverse-transcribed after the genomic DNAs were removed using a reverse transcription kit (Takara, Tokyo, Japan). The cDNA product was stored at –20°C. For real-time PCR, a 10 μl reaction mixture containing 50 ng cDNA was used. The primer sequences were:

β-actin (mouse)
Forward: 5′-TGCTGTCCCTGTATGCCTCT-3′
Reverse: 5′-TTGATGTCACGCACGATTTC-3′
Nogo-C (mouse)
Forward: 5′-CAGAAGAAACGTTGGAAGGACA-3′
Reverse: 5′-ATAGTCACAGAGAGCAGGGC-3′

### Immunohistochemical Staining Assay

Nerves were fixed with 4% paraformaldehyde and embedded with paraffin wax. The sections were perfused in 3% H_2_O_2_ to clear endogenous peroxidase and microwaved in sodium citrate buffer (1 mM, pH 6). The slides were blocked in 1% BSA for 30 min at 37°C, probed with anti-Nogo-C antibody (1:100) overnight at 4°C, and then a horseradish peroxidase-conjugated secondary antibody at 37°C for 30 min.

### Immunofluorescence

The distal sciatic nerve was removed and placed in 4% paraformaldehyde for 10 min, and permeabilized with 0.5% Triton-100 for 15 min. Nerves were then blocked with 5% goat serum for 30 min, incubated with indicated S100β (1:500) (66616-1-Ig, proteintech, Wuhan, China) at 4°C overnight, and incubated with Alexa-fluor 488 goat-anti-mouse IgG, 1:200 for 1 h at room temperature. 4,6-diamidino-2-phenylindole 303 (DAPI, Sigma-Aldrich) was used to visualize the nuclei. Images were captured on a laser scanning confocal microscopy (TCS SP5 II, Leica).

### Cell Death Assay

Cell apoptosis was determined by TUNEL (terminal deoxyribonucleotidyl transferase-mediated dUTP-digoxigenin nick-end labeling) assay using the *in situ* Cell Death Detection Kit (Roche, Basel, Switzerland).

### Cell Proliferation

Cells were seeded into 96-well plates at a density of 1 × 104 cells/well. Cell Counting Kit 8 (CCK-8) solution (Dojindo, Tokyo, Japan) was added into each well, followed by a 2 h incubation. The absorbance, or optical density (OD), was measured at 450 nm with a microplate reader (Bio-Rad).

### Statistical Analysis

All data are presented as mean ± SEM. Statistical significance was analyzed via *t*-test or one-way ANOVA. *P* < 0.05 was considered statistically significant. GraphPad Prism 8 software (GraphPad Software, La Jolla, CA, United States) was used for all statistical analyses.

## Results

### Nogo-C Was Elevated at the Distal End of the Injured Sciatic Nerve

Nogo-C expression increased 7–14 days after the injury (Figures 1A–C). In addition, immunohistochemical staining (Figure 1D) was consistent with the Western blot and RT-PCR results. Nogo-C expression increased in the distal end of the injured sciatic nerve in mice, suggesting that Nogo-C may be involved in peripheral nerve repair.

**FIGURE 1:** Nogo-C is upregulated in crush mouse sciatic nerves. **(A,B)** Western blot and mean data showing Nogo-C protein expression in sham and crush mouse sciatic nerves 7 and 14 days after operation; *n* = 3 mice per group. **(C)** RT-PCR showing Nogo-C mRNA levels in sham and crush mouse sciatic nerves 7 and 14 days after the operation; *n* = 4 mice per group. *P < 0.05, **P < 0.01 vs. sham group. **(D)** Nogo-C immunohistochemical staining of sham (left) and crush mouse sciatic nerves 7 days (right, a: proximal; b: distal) after the operation.

### Nogo-C Knockout Promoted the Regeneration of Injured

In order to understand the role of Nogo-C in sciatic nerve injury repair, a Nogo-C^–/–^ mouse model was established (Figure 2A). No differences in sciatic nerve index (SFI) were observed between the 8 weeks-old Nogo-C^–/–^ and WT group (Figures 2B,C). After injury, postoperative dynamic observation showed that the SFI of the Nogo-C^–/–^ group was higher than the WT group 7–28 days after the injury.

**FIGURE 2:** Nogo-C knockout promotes sciatic nerve regeneration. **(A)** Western blot shows the Nogo-C protein level in sciatic nerves from WT and Nogo-C^–/–^ mice. Nogo-C^–/–^ mice show no significant expression of Nogo-C in the sham and crush groups. **(B,C)** Sciatic Function Index between WT and Nogo-C^–/–^ mice before (–1 day) and after sciatic nerves injury; *n* = 4 mice per group. **(D)** A typical example of semi-thin sections of WT and Nogo-C^–/–^ tibial nerves 2 weeks after crush injury and sham; scale bar = 20 μm. **(E)** Mean number of axons in tibial nerves; *n* = 6 mice per group. **(F)** Representative Toluidine blue-stained ultrathin section of WT and Nogo-C^–/–^ tibial nerves 2 weeks after crush injury and sham; scale bar = 5 μm. **(G)** Myelin thickness relative to axon diameter was quantified in cross-sections of uninjured (sham) and injured (crush) tibial nerves of four WT and four Nogo-C^–/–^ mice 2 weeks after crush injury and illustrated as a scatter plot. 50 axons and myelin sheath were measured from each nerve and shown in the plot. There were significant differences (*p* < 0.001) between WT and Nogo-C^–/–^ nerves at 2 weeks of regeneration and no difference between sham groups. ^$$^*P* < 0.01, ^$$$^*P* < 0.001 vs. WT sham, *P < 0.05, ***P < 0.001 vs. Nogo-C^–/–^ sham, ^##^*P* < 0.01, ^###^*P* < 0.001 vs. WT crush.

Semi-thin and ultra-thin sections of the tibial nerve were prepared 14 days after surgery. The semi-thin sections (Figures 2D,E) showed no difference in the number of tibial nerves between WT and Nogo-C^–/–^ mice in the sham operation group and the number of distal tibial nerves in the Nogo-C^–/–^ group was higher than in the WT controls 14 days after nerve injury, and both were higher than the corresponding sham groups. In addition, the myelination of regenerating axons was observed with electron transmission microscopy 14 days after surgery (Figures 2F,G). No difference in the thickness of myelin sheaths between the Nogo-C^–/–^ and WT groups was observed. The ratio of myelin thickness/axon diameter of the distal regenerating nerves in Nogo-C^–/–^ mice was increased compared with WT mice, indicating that knocking out the Nogo-C gene favored remyelination. These results suggested that the growth and development of the sciatic nerve were not affected by Nogo-C gene knockout in mice, and the regeneration rate after nerve injury was accelerated.

### Nogo-C Promoted Schwann Cell Apoptosis

Nogo-C protein expression was increased in neonatal rat Schwann cells transfected with adenovirus containing Nogo-C cDNA (Ad-Nogo-C) (Figures 3A,B). Overexpression of Nogo-C increased Schwann cell apoptosis. As shown by TUNEL staining, apoptosis in Ad-Nogo-C-expressing cells was higher than control cells (Figures 3C,D). In addition, cell apoptosis at the distal end of the nerve was observed 7 days after nerve injury, and Nogo-C knockout can significantly reduce apoptosis after nerve injury (Figures 3E,F). The protective effect of Nogo-C knockout on Schwann cell apoptosis was confirmed by Western blot analysis of the distal end of the injured nerve (Figures 3G,H). In the process of neural injury-induced Schwann cell apoptosis, Bcl-2 inhibited cell apoptosis and BAX promoted cell apoptosis. In addition, the ratio of Bcl-2/BAX protein expression in the distal end of the injured nerve in Nogo-C^–/–^ mice was twice as high as the WT group. Therefore, our results demonstrated that Nogo-C induced Schwann cell apoptosis, while Nogo-C knockout reduced Schwann cell apoptosis.

**FIGURE 3:** Nogo-C regulates cardiomyocyte apoptosis. **(A,B)** Western blot showing Nogo-C protein expression in rat neonatal Schwann cells transfected with Ad-Nogo-C at 75 MOI or Ad-lacz for 48 h; *n* = 3 independent experiments. **(C,D)** TUNEL staining showing apoptotic rates of Schwann cells transfected with Ad-Nogo-C or Ad-lacz; *n* = 6 independent experiments. Scale bar = 25 μm. **P < 0.001, ***P < 0.001 vs. Ad-lacz cells. **(E,F)** TUNEL staining showing apoptotic cells in sham and crushed (7 days after the operation) sciatic nerves from WT and Nogo-C^–/–^ mice. *n* = 4 mice. Scale bar = 25 μm. **(G,H)** western blot and average data showing BAX Bcl-2 and MPZ protein levels in sham and crushed sciatic nerves from WT and Nogo-C^–/–^ mice; *n* = 3 mice for each group. ^$$$^*P* < 0.001 vs. WT sham, *P < 0.05, ***P < 0.001 vs. Nogo-C^–/–^ sham, ^###^*P* < 0.001 vs. WT crush.

### Nogo-C Inhibited Schwann Cell Dedifferentiation

Dedifferentiation of Schwann cells is vital to the repair of injured nerve. In the dedifferentiation process, Krox-20 is downregulated and c-Jun is upregulated in Schwann cells. Dedifferentiated Schwann cells participate in a series of processes, including demyelination, to promote nerve regeneration. Western blot analysis showed that when Nogo-C was overexpressed in neonatal rat Schwann cells via adenovirus-mediated gene transfer, the expression of c-Jun and GFAP decreased by 50% and the expression of Krox-20 and MPZ was up-regulated twofold compared with the control group. The ratio of c-Jun/Krox-20 was also significantly reduced to 1/4 of the control group (Figures 4A–C). These results suggest that Nogo-C inhibited the dedifferentiation of Schwann cells. In addition, proliferative capacity is an altered feature of Schwann cells after dedifferentiation. We used cck-8 to detect the proliferative capacity of primary Schwann cells. When Nogo-C was overexpressed, the ability of Schwann cells to proliferate significantly decreased when compared with the control group from the third day (Figure 4D). *In vivo*, myelination in the distal tibial nerves was observed 7 days after injury by TEM. The number of residual myelin in Nogo-C^–/–^ mice was less than that in WT mice (Figures 4E,F). We also investigated Mpz clearance by western blot 7 days after nerve injury, We found that MPZ expression in the distal end of the injured nerve on day 7 post-injury was significantly less than in the sham group. MPZ expression in the crush-Nogo-C-knock group was significantly lower than that in the crush-WT group (Figures 3G,H). This suggest that myelin disintegration at the distal end of the injured nerves, which is mainly regulated by dedifferentiated Schwann cells 7 days after crush, was faster in Nogo-C^–/–^ mice than WT mice.

**FIGURE 4:** Nogo-C inhibited Schwann cell dedifferentiation. **(A–C)** Western blot and average data of protein levels of dedifferentiation proteins in Schwann cells transfected with Ad-Nogo-C or Ad-Lacz for 48 h. **(D)** CCK-8 assays of Schwann cells transfected with Ad-Nogo-C or Ad-Lacz for 48 h; *n* = 3 independent experiments. *P < 0.05, ***P < 0.001 vs. Ad-LacZ transfected cells. **(E)** Representative Toluidine blue-stained ultrathin section of sham and crushed (7 days after operation) tibial nerves from WT and Nogo-C^–/–^ mice; scale bar = 5 μm. **(F)** Average number of axons in each field of view from tibial nerves; *n* = 6 mice per group. ^$^*P* < 0.05 vs. WT sham, ***P < 0.001 vs. Nogo-C^–/–^ sham, ^###^*P* < 0.001 vs. WT crush.

## Discussion

Members of the Nogo gene family play an important role in various physiological and pathological processes and their functions in the CNS have been well documented. The results from our study suggest that Nogo-C is closely related to peripheral nerve repair after peripheral nerve injury, as evidenced by the following findings: (1) Nogo-C expression was increased in the distal end of the injured sciatic nerve; (2) Nogo-C knockout accelerated the repair of injured sciatic nerve and reduced the number of apoptotic cells in the injured nerve lesions; and (3) overexpression of Nogo-C simultaneously promoted Schwann cell apoptosis and inhibition of dedifferentiation.

To investigate the effect of Nogo-C on peripheral nerve repair, we generated a Nogo-C knockout mouse model. The sciatic nerve was crushed in Nogo-C^–/–^ and WT mice to examine the subsequent nerve recovery. Evaluation of sciatic nerve repair showed that the number of regenerated nerve fibers in the distal end of the injured nerves increased in the Nogo-C^–/–^ and WT mice 14 days after sciatic nerve injury compared with the sham operation groups. However, diameter and myelin thickness were reduced compared with the sham operation group. This was consistent with previous studies (Li et al., 2003). We believed this is due to the formation of a large number of side branches during nerve regeneration. Comparison between groups showed that the ratio of regenerated nerve fibers in the Nogo-C^–/–^ experimental/sham operation mice increased compared with WT mice, indicating that Nogo-C gene knockout was beneficial to axonal budding. This may serve as a new intervention target to improve the prognosis of neurotransplantation.

Schwann cells are essential regulators of peripheral nerve repair (Huang et al., 2016), sensing and responding to a nerve injury within hours (Martini et al., 2008). First, mature and differentiated myelinating Schwann cells transform into repairing Schwann cells, which are suitable for nerve repair. This process is known as Schwann cell dedifferentiation, which involves phenotypic transition and the reversal of myelination. During Schwann cell demyelination, pre-myelinating Schwann cell-specific markers, such as GFAP, are up-regulated. In addition, myelination-related genes are down-regulated, including the key myelin transcription factor Krox20 [26]. Importantly, c-Jun, which promotes the down-regulation of myelination and is required for the normal activation of repair, is rapidly upregulated. In the present study, we explored the effect of Nogo-C on Schwann cells. Nogo-C was overexpressed in isolated primary Schwann cells. Nogo-C significantly downregulated the expression of c-Jun and GFAP, and significantly up-regulated Krox20 in Schwann cells. This process is the opposite of Schwann cell demyelination. Therefore, Nogo-C could affect nerve repair by inhibiting the dedifferentiation of Schwann cells. In addition, Schwann cells promote axon regeneration via demyelination in the distal end of the injured nerve. The distal demyelination reached its peak 7 days after the nerve injury. TEM of the distal nerve sections 7 days after the nerve injury showed that residual myelination in the Nogo-C^–/–^ group was significantly less than the WT group, indicating that the demyelination in the Nogo-C^–/–^ group was faster. This confirmed that Nogo-C inhibits Schwann cell dedifferentiation and demyelination. However, whether other molecular mechanisms are involved in the inhibitory demyelination effect of Nogo-C, and whether Nogo-C may affect other Schwann cells nerve repair factors requires further elucidation.

Nogo-C promotes the apoptosis of HEK293 cells (Chen et al., 2006) and cardiomyocyte after myocardial infarction (Jia et al., 2016). Therefore, we speculated that Nogo-C could also mediate Schwann cell apoptosis. In the present study, cell apoptosis of the distal nerve was observed 7 days after the nerve injury, and the number of apoptotic cells in the distal nerve was significantly increased in the experimental group compared with the sham group. This finding is consistent with previous results (Grinspan et al., 1996; Trachtenberg and Thompson, 1996) that demonstrated a large amount of apoptotic Schwann cells following axon transection after the peripheral nerve injury and the up-regulation of Bcl-2 protects Schwann cells from apoptosis. In the present study, TUNEL staining showed that the number of apoptotic cells in the distal nerve of the Nogo-C^–/–^ group was significantly lower than that in the WT group. Importantly, western blot showed that Bcl-2 protein expression in the injured nerves was significantly increased in the Nogo-C^–/–^ group compared with that in the WT group, suggesting that Nogo-C knockout protected Schwann cells from apoptosis after nerve injury. Furthermore, Nogo-C overexpression in Schwann cells increased the number of apoptotic cells, suggesting Nogo-C could induce Schwann cell apoptosis. These results suggest that increased Nogo-C expression in local lesions after sciatic nerve injury could delay the regeneration of injured nerves by promoting Schwann cell apoptosis.

## Conclusion

Our study provides evidence that Nogo-C is upregulated following sciatic nerve injury and Nogo-C knockout could promote the regeneration of injured sciatic nerves and recovery of limb motor function *in vivo*. In addition, Nogo-C knockout reduced Schwann cell apoptosis around injured nerves. The overexpression of Nogo-C in Schwann cells promotes Schwann cell apoptosis and inhibits Schwann cell dedifferentiation. Our data suggests that Nogo-C could inhibit peripheral nerve regeneration by promoting Schwann cell apoptosis and inhibition of Schwann cell dedifferentiation. Therefore, Nogo-C and associated pathways could be potential therapeutic targets for peripheral nerve repair.

## Data Availability Statement

The datasets during and/or analyzed during the current study available from the corresponding author on reasonable request.

## Ethics Statement

The animal study was reviewed and approved by Animal Protection Committee of Peking University Health Science Center.

## Author Contributions

BJ, WH, MZ, and TW: conceptualization. BJ and YW: methodology. BJ, YW, and PZ: software and investigation. BJ: writing—original draft. MZ and TW: writing—review and editing, supervision, and funding acquisition. All authors read and approved the final manuscript.

## Conflict of Interest

The authors declare that the research was conducted in the absence of any commercial or financial relationships that could be construed as a potential conflict of interest.

## Abbreviations

GFAP: glial fibrillary acidic protein
MAG: myelin-associated glycoprotein
MBP: myelin basic protein
NGF: nerve growth factor
SFI: sciatic function index
TEM: transmission electron microscopy
TS: total spreading.
